# The Effects of Sequential Ventilation Therapy on Blood Gas Indexes, Pulmonary Function Indexes, Clinical Efficacy, and Safety in Patients with Severe Cor Pulmonale

**DOI:** 10.1155/2022/3618592

**Published:** 2022-10-07

**Authors:** Jianmeng Cheng, Xingxing Dou, Na Zhao

**Affiliations:** ^1^Respiratory Department, Lianshui County People's Hospital, Lianshui 223400, China; ^2^Department of Rehabilitation Medicine, The Affiliated Huai'an Hospital of Xuzhou Medical University, The Second People's Hospital of Huai'an, Huaian 223002, China; ^3^Department of Respiratory Medicine, Hongze District People's Hospital, Huaian 223100, China

## Abstract

As a heart disease caused by pulmonary arterial hypertension, pulmonary heart disease has a high incidence and poor clinical prognosis in the elderly. Including mechanical ventilation in the current clinical treatment of cor pulmonale, with the development of medical technology, traditional invasive mechanical ventilation has been pointed out to have certain clinical limitations, so new invasive and noninvasive sequential ventilation treatments are gradually being used. Applied in clinical practice, this article selected 96 patients with severe cor pulmonale in our hospital from January 2020 to May 2021 as the research object and conducted a randomized prospective study. The experimental results show that the two general methods can improve the blood gas index and pulmonary function index of patients with heart disease and pulmonary dysfunction, but the improvement of the above indexes by the sequence of action of gas therapy is better than that of conventional invasive mechanical ventilation.

## 1. Introduction

Pulmonary heart disease is a common chronic respiratory disease in middle-aged and elderly people, which is accompanied by pulmonary function and cardiac dysfunction as the main clinical symptoms, which greatly affects the prognosis, survival, and quality of life [1]. In clinical practice, cor pulmonale is mainly divided into acute cor pulmonale and chronic cor pulmonale, and the causes of both are different. The main cause of acute cor pulmonale is the sharp increase of pulmonary artery pressure in a short period of time. When the right ventricle cannot adapt to the trend of a sudden increase in pulmonary artery pressure, right ventricle dilatation and compensatory disorder will occur [2]. The main cause of chronic cor pulmonale is pulmonary interstitial and vascular fibrosis caused by chronic obstructive pulmonary disease, which leads to symptoms such as cardiac dysfunction and heart failure caused by increased right ventricular load [3].

Although the causes of cor pulmonale are different, they jointly affect the heart function and lung function of patients, lead to respiratory tract infection and increase the risk of respiratory failure and heart failure. Therefore, safe and effective treatment has always been the common appeal of respiratory experts and such patients [4]. Clinical practice shows that correct hypoxia is a key link in the process of treatment of cor pulmonale, which may increase the alveolar ventilation through mechanical ventilation, improve ventilation function, and thus improve the ability to work in patients with cardiopulmonary. However, it still has the characteristics of difficult weaning and a high incidence of ventilator-associated pneumonia, which limits its clinical application [5, 6]. With the continuous support of new technologies, invasive and noninvasive sequential ventilation therapy has been gradually applied in clinical practice, but its clinical efficacy and safety have not been elucidated by too many studies. Therefore, this study selects 96 patients with severe cor pulmonale as the research object to observe the clinical efficacy and safety of sequential ventilation therapy. The results show that the incidence of adverse reactions is significantly reduced.

The rest of this paper is organized as follows: Section 2 discusses related work, followed by focusing on general information and treatment methods in Section 3. The comparison of various indicators and changes are discussed in Section 4.  Section 5 concludes the paper with a summary.

## 2. Related Work

Severe cor pulmonale high rates of respiratory failure in older adults, lung function in patients with severe damage, air-breathing difficulties, leading to a lack of oxygen or with CO_2_ retention, concurrent mental nerve symptoms, pulmonary encephalopathy or gastrointestinal bleeding, triggered a series of physiological function disorder, serious and even death, serious influence on patients' daily life [7]. At present, invasive mechanical ventilation was a widely used method for the clinical treatment of respiratory failure of severe cor pulmonale, but its improvement of cardiac function and blood rheology of patients could not meet the expectations [8]. Gen-non-invasive sequential gas ventilation was a new treatment method developed from invasive mechanical ventilation. It could be used for noninvasive ventilation treatment of patients with respiratory failure and infection control after initial treatment, replacing nasal and oral mask endotracheal intubation [9]. However, there were few clinical studies on this treatment. Therefore, a prospective trial was conducted to further explore the clinical efficacy of sequential ventilation therapy.

By observing the ventilation time of the two groups, it was shown that the invasive ventilation time and total ventilation time of the study group were significantly shorter than those of the control group, indicating that sequential ventilation therapy could reduce the time of tracheal intubation, thereby reducing the invasive ventilation time [10]. In addition, the comparison of blood gas indexes at different time periods before and after treatment showed that the PH changes of the two groups were consistent and had no significant difference after treatment, indicating that both treatment methods could better maintain PH stability [11]. After different treatments, the blood oxygen value of the two groups increased, while the blood carbon dioxide value decreased, and the improvement of PaCO_2_ and PaO_2_ in the study group was significantly better than that in the control group. The analysis of the results suggested that PaCO_2_ was the pressure or tension caused by dissolved carbon dioxide in the blood. It is commonly used in clinical practice to judge the type of respiratory failure, whether there was a respiratory acid-base imbalance, compensatory reaction of metabolic acid-base imbalance, or alveolar ventilation [12].

When the PaCO_2_ value of patients with severe cor pulmonale increased, it indicated insufficient lung ventilation and CO_2_ retention, and patients might have symptoms such as breathing and sleep disorders. However, sequential ventilation therapy reduced the time of tracheal intubation, so it caused less damage to the lungs and could better help patients with pulmonary ventilation [13]. Sequential ventilation therapy could improve spontaneous breathing, reduce airway resistance and improve alveolar oxygenation function as soon as possible, so the recovery of PaO_2_ was significantly better than that of invasive mechanical ventilation [14].

## 3. General Information and Treatment Methods

### 3.1. General Information

This article selected 96 patients with severe cor pulmonale in our hospital from January 2020 to May 2021 as the research object and conducted a randomized prospective study. They are randomly divided into the study group (*n* = 48) and the control group (*n* = 48). All the patients are coded from 1 to 96 and put into EXCEL. The even number of patients is included in the study group, and the odd number of patients is included in the control group. All patients have the right to know and consent to the treatment used in the study and are aware of possible adverse reactions [15]. Patients with poor physical tolerance, congenital immune dysfunction, and poor treatment compliance are excluded.

### 3.2. Treatment Methods

Both groups are given the same routine treatment operations, including anti-infection, airway dilation, correction of water and electrolytes, and incision of tracheal intubation is connected to an external ventilator. On this basis, the control group is treated with invasive mechanical ventilation in the supine position, with a tidal volume of 8–10 ml/kg and a breathing reserve (BR) of 10–20 times/min in synchronized intermittent mandatory ventilation (SIMV) mode. Pressure support ventilation mode is adopted after the patient's respiratory function improved significantly. The patients in the study group are treated with invasive and noninvasive sequential ventilation. The patients are in the supine position, the tidal volume in SIMV mode is 8–10 ml/kg, and the BR is 10–20 times/min. After the respiratory function is significantly improved, the tracheal tube is removed and the noninvasive ventilator is used for noninvasive mask double-level positive pressure ventilation. Adjust BR to 12 to 20 beats/min, inspiratory pressure to 14 to 18cm H_2_O, and inspiratory pressure to 4 to 6cm H_2_O. Both groups are treated for 1 week [16].

A blood gas analyzer is used to detect the blood gas parameters before treatment (T0), 3 days after treatment (T1), and 1 week after treatment (T2), including PH, PaO_2,_ and PaCO_2_.

Before and after treatment, the percentage of forced expiratory volume In 1s (FEV1) to the predicted value, the ratio of FEV1 to forced vital capacity (FVC) (FEV1/FVC), and peak expiratory flow (PEF) rate is measured. Vital capacity values are measured with a Jester spirometer.

The improvement of symptoms such as respiratory failure and dyspnea after treatment is considered a significant effect. Improvement in clinical symptoms is considered as effective. No significant improvement in clinical symptoms after 1 week of treatment is considered to be ineffective. The clinical effective rate is equal to (significant effective + ineffective)/the number of people a ×100%.

### 3.3. Statistical Treatment

SPSS 25.0 statistical software is used for data analysis. If the data obey normal distribution and homogeneity of variance after the normal test, it is expressed as mean ± standard deviation. One-way ANOVA is used to analyze the data between multiple groups, repeated measurement analysis is used to analyze multiple time points within the same group, and a spherical test is performed [17]. Descriptive statistical analysis is performed by percentage, and the *x*2 test is used. Kaplan–Meier method is used to observe the incidence of adverse reactions. *P* < 0.05 is considered a significant difference.

## 4. Comparison of Various Indicators and Changes

### 4.1. Comparison of Baseline Data between the Two Groups

Table 1 shows the clinical baseline data of the three groups. It is clearly evident from Table 1 that there is no significant difference in baseline data between the two groups, and there is no interference due to age, gender, and other factors.

### 4.2. Comparison of Ventilation Indexes

Table 2 shows the comparison of ventilator-related indicators. It is clearly evident from Table 2 that the duration of invasive ventilation in the control group is around 6.4.

Figure 1 shows the comparison of ventilator-related indicators. It is clearly evident from Figure 1 that the duration of invasive ventilation, total ventilation time, and length of hospital stay in the study group are significantly lower than those in the control group.

### 4.3. Changes in Blood Gas Indexes before and after Treatment

Table 3 shows the changes in blood gas indexes before and after treatment. It is clearly evident from Table 3 that the pH value of the two groups increased to a certain extent after treatment, but there is no significant difference between the two groups. In the two groups after treatment and through different ways PaCO_2_ is declining.

Figure 2 shows the changes in blood gas indexes before and after treatment. It is clearly evident from Figure 2 that the research in all time points after the treatment levels of indicators are superior to the control group, and it shows that both methods have a certain effect on improving the blood gas index of patients with heart disease and lung disease, but the sequential treatment of improving blood gas has a more significant effect.

### 4.4. Changes in Lung Function before and after Treatment

Table 4 shows the lung function changes before and after treatment. It is clearly evident from Table 4 that the lung function of the two groups is improved to varying degrees after different treatments, and the improvement of the study group is significantly better than that of the control group.

### 4.5. Comparison of Clinical Effective Rate

Table 5 shows the comparison of clinical response rates. It is clearly evident from Table 5 that although there is no significant difference in clinical efficacy between the two groups, the number of patients with significant efficacy in the study group is significantly higher than that in the control group.

Figure 3 shows the comparison of clinical response rates. It is clearly evident from Figure 3 that sequential ventilation therapy is more effective in improving the clinical symptoms of patients with cor pulmonale.

### 4.6. Comparison of the Incidence of Adverse Reactions

Figure 4 shows the comparison of the incidence of adverse reactions. It is clearly evident from Figure 4 that during the one-week treatment period, a total of 6 patients (12.50%) in the study group have adverse reactions, while 14 patients (29.17%) in the control group have adverse reactions. The Kaplan–Meier curve shows that there is a significant difference in the incidence of adverse reactions between the two groups. The safety of sequential ventilation is significantly better than that of traditional mechanical ventilation (*x*2 = 4.307, *P*=0.038).

## 5. Conclusion

This study further compares the clinical efficacy and safety of the two treatment methods. The results show that there is almost no difference in the clinical efficacy of the two treatment methods, but the order of clinical cases treated by Qi therapy is significantly improved than that of the control group, and the incidence of adverse reactions is significantly reduced, further indicating that it has high clinical value and safety. In conclusion, sequential ventilation therapy can effectively improve blood gas indexes and pulmonary function indexes in patients with severe cor pulmonale, improve clinical efficacy, reduce adverse reactions, and has high clinical application value.

## Figures and Tables

**Figure 1:** Comparison of ventilator-related indicators: (a) duration of invasive ventilation; (b) total ventilation time; (c) the hospitalization time.

**Figure 2:** Changes in blood gas indexes before and after treatment: (a) PH; (b) Paco_2_; (c) PaO_2_.

**Figure 3:** Comparison of clinical response rates: (a) control group; (b) study group.

**Figure 4:** Comparison of the incidence of adverse reactions.

**Table 1:** Clinical baseline data of the three groups.

Group	*n*	Age (years)	Gender		BMI (kg/m^2^)
			Man	Woman	
Control group	48	56.46 ± 6.50	29 (60.42)	19 (39.58)	24.28 ± 1.38
Study group	48	57.38 ± 6.76	27 (56.25)	21 (43.75)	24.22 ± 1.34
*t*/*x*2		−0.677	0.171		0.199
*P*		0.500	0.679		0.843

**Table 2:** Comparison of ventilator-related indicators.

Group	*n*	Duration of invasive ventilation (d)	Total ventilation time (d)	The hospitalization time (d)
Control group	48	6.40 ± 1.14	15.50 ± 1.78	19.83 ± 2.81
Study group	48	4.81 ± 1.44	10.13 ± 1.55	14.52 ± 2.22
*T*		5.986	15.795	10.279
*P*		< 0.001	< 0.001	< 0.001

**Table 3:** Changes in blood gas indexes before and after treatment.

Group	*n*	pH		
		T0	T1	T2
Control group	48	7.23 ± 0.04	7.29 ± 0.03	7.38 ± 0.05ab
Study group	48	7.23 ± 0.05	7.30 ± 0.03	7.37 ± 0.05ab
*T*		−0.169	−1.118	1.393
*P*		0.866	0.266	0.167
		PaCO_2_ (mmHg)		

		T0	T1	T2
Control group	48	65.10 ± 3.32	63.42 ± 4.06	55.46 ± 3.90ab
Study group	48	64.90 ± 3.50	61.36 ± 3.88a	53.39 ± 3.48ab
*T*		0.297	−2.533	−2.756
*P*		0.767	0.013	0.007
		PaO_2_ (mmHg)		

		T0	T1	T2
Control group	48	64.24 ± 3.28	71.86 ± 3.47a	76.10 ± 3.94ab
Study group	48	65.34 ± 3.79	74.30 ± 3.70a	80.65 ± 4.22ab
*T*		−1.520	3.344	5.465
*P*		0.132	0.001	＜ 0.001

**Table 4:** Lung function changes before and after treatment.

Group	*n*	FEV1 (%)		FEV1/FVC (%)		PEF (L/min)	
		Before	After	Before	After	Before	After
Control group	48	53.45 ± 3.97	58.01 ± 4.34a	51.34 ± 4.18	58.16 ± 3.93a	260.19 ± 23.75	320.15 ± 30.24a
Study group	48	53.78 ± 3.98	67.26 ± 3.69a	52.05 ± 3.92	63.84 ± 4.25a	267.19 ± 24.44	397.05 ± 28.79a
*T*		−0.408	−11.247	−0.866	−6.790	−1.422	−12.761
*P*		0.684	< 0.001	0.389	< 0.001	0.158	<0.001

**Table 5:** Comparison of clinical response rates.

Group	*n*	Significant curative effect	Effective	Invalid	Effective rate
Control group	48	18 (37.50)	19 (39.58)	11 (22.92)	37 (77.08)
Study group	48	29 (60.42)	11 (22.92)	8 (16.67)	40 (83.33)
*x*2		5.044	3.103	0.591	0.591
*P*		0.025	0.078	0.442	0.442

## Data Availability

The simulation experiment data used to support the findings of this study are available from the corresponding author upon request.
